The article "CDKL5 promotes proliferation, migration, and chemotherapeutic drug resistance of glioma cells via activation of the PI3K/AKT signaling pathway" was retracted in 2024. Reasons: plagiarized images; overlap with other authors' work; unreliable data; unreliable results or conclusions.

# CDKL5 promotes proliferation, migration, and chemotherapeutic drug resistance of glioma cells via activation of the PI3K/AKT signaling pathway

**DOI:** 10.1002/2211-5463.12780

**Published:** 2020-01-21

**Authors:** Zhenfu Jiang, Tongtong Gong, Hong Wei

**Affiliations:** ^1^ Department of Neurosurgery The Second Hospital of Dalian Medical University China; ^2^ Department of Neurosurgery Dalian Medical University China; ^3^ Department of Pathology The First Affiliated Hospital of Dalian Medical University China

**Keywords:** CDKL5, drug resistance, glioma, migration, PI3K, AKT

## Abstract

Gliomas, the most prevalent cancer in the central nervous system, are characterized by high morbidity and mortality, emphasizing the need to understand their etiology. Here, we report that cyclin‐dependent kinase‐like 5 (CDKL5) is highly expressed in gliomas, and CDKL5 overexpression promotes invasion, proliferation, migration and drug (β‐lapachone) resistance of glioma cells. *In vitro*, CDKL5 overexpression enhanced invasion, growth and migration of glioma cells, and stimulated the phosphoinositide 3‐kinase (PI3K)/AKT axis. Furthermore, CDKL5 overexpression *in vivo* promoted glioma proliferation, whereas CDKL5 knockdown had opposing effects. The effect of CDKL5 on drug resistance was eliminated if the PI3K/AKT axis was suppressed, and cisplatin combined with the PI3K/AKT suppressor XL147 remarkably prohibited proliferation in xenografts overexpressing CDKL5. Collectively, our findings suggest that CDKL5 acts through the PI3K/AKT axis in glioma cells, and indicate a possible role for CDKL5 in glioma therapy.

## Graphical abstract

Cyclin‐dependent kinase‐like 5 promotes the proliferation, migration, drug resistance and invasion of glioma cells, which contributes to glioma growth *in vivo* by stimulating the phosphoinositide 3‐kinase/AKT axis. This research suggests that cyclin‐dependent kinase‐like 5 may have potential in the assessment of clinical outcome and treatment of gliomas.

**Abbreviations**
β‐lap: β‐lapachone
CDKL5: cyclin‐dependent kinase‐like 5
β‐lap: β‐lapachone
CDKL5: cyclin‐dependent kinase‐like 5
DMEM: Dulbecco’s modified Eagle’s medium
FC: flow cytometry
IHC: immunohistochemistry
MTT: 3‐(4,5‐dimethylthiazol‐2‐yl)‐2,5‐diphenyl‐tetrazolium bromide
KD: knockdown
PI3K: phosphoinositide 3‐kinase
SEM: standard error of the mean
TBS: Tris‐buffered saline
WB: western blotting

As the most prevalent cancer in the central nervous system because of the noticeable incidence rate, fast relapse and limited survival 1, gliomas are characterized by persistent growth, reinforced migration and invasion, and multiple molecular and cytogenetic aberrances 2. Standard glioma therapy consists of surgery 3 before radiotherapy 4 and chemotherapy 5. Nevertheless, drug resistance is a difficult challenge to overcome 6. Despite progress in malignancy therapy, the clinical outcome of patients with glioma is far from satisfactory, and <5% of patients survive for 5 years after diagnosis 7. Furthermore, the understanding of the molecular etiology of gliomas is insufficient 8. Consequently, it is urgent to elucidate the etiology and to recognize innovative targets for the treatment of gliomas 9, 10.

The article "CDKL5 promotes proliferation, migration, and chemotherapeutic drug resistance of glioma cells via activation of the PI3K/AKT signaling pathway" was retracted in 2024. Reasons: plagiarized images; overlap with other authors' work; unreliable data; unreliable results or conclusions.

As a serine/threonine kinase, cyclin‐dependent kinase‐like 5 (CDKL5) was recognized via transcriptional mapping research focusing on the recognition of genes that brought about illness in Xp22 region 1 11. The recognition of CDKL5 mutations in patients suffering from the Hanefeld variant of Rett syndrome of infantile epileptic encephalopathy in the early stage implicated the activity of CDKL5 in the human cerebra 12, 13, 14. Accordingly, two present murine models with CDKL5 knockouts featured reduced studying and recollection, characteristics resembling autism, and motor defects that complied with some aspects of clinical spectrum in patients displaying CDKL5 mutations 15, 16. CDKL5/CDKL5 gene transcription is prevalent, and proteins can be examined in most tissues and cells, not only in the nucleus but also in the cytoplasm 17. Because the expression of CDKL5 reaches peak levels in the cerebra because of obvious cerebra‐related activities, most research has aimed at the neuronal influence of CDKL5 18, 19, 20. Nevertheless, the understanding of its influence on gliomas is insufficient.

We investigated CDKL5 expression in gliomas and evaluated CDKL5 functions in the modulation of the biological activities of gliomas. Moreover, the promising etiology of gliomas was recognized.

## Materials and methods

### Cell lines and tissue samples

The human glioma cell lines U87 (glioblastoma of unknown origin, BNCC337885) and U251 were acquired from the Type Culture Collection of the Chinese Academy of Sciences (Shanghai, China) and subsequently preserved in 5% CO_2_ in Dulbecco’s modified Eagle’s medium (DMEM; HyClone, St. Louis, MO, USA) containing 10% FBS (Gibco, Billerica, MA, USA) at 37 °C.

Twenty‐seven patients received clinical and histological diagnoses of gliomas at The First Affiliated Hospital of Dalian Medical University. Fully written informed consent was acquired, and our research was approved by the Ethics Committee of The First Affiliated Hospital of Dalian Medical University. The study methodologies conformed to the standards set by the Declaration of Helsinki. Cerebral tissue specimens were acquired from five patients who had encountered intracerebral hemorrhage. All samples were kept at −80 °C.

The article "CDKL5 promotes proliferation, migration, and chemotherapeutic drug resistance of glioma cells via activation of the PI3K/AKT signaling pathway" was retracted in 2024. Reasons: plagiarized images; overlap with other authors' work; unreliable data; unreliable results or conclusions.

### Immunohistochemistry

Paraffin slices (5 μm) of glioma and normal cerebral tissues were subjected to dehydration using a graded concentration series of ethanol before incubation in H_2_O_2_ with 1% BSA in Tris‐buffered saline (TBS). The specimens were incubated overnight with murine IgG isotype antibody or mouse anti‐human CDKL5 IgG at 4 °C in a humid chamber. The slices were covered with goat anti‐mouse IgG antibody conjugated with peroxidase (SP‐9002; Golden Bridge International, Inc., Beijing, China) after three washes with TBS.

### RNA isolation and quantitative PCR

TRIzol (Life Technologies, St. Louis, MO, USA) was used to isolate total RNA from tissues, which was purified using the RNeasy Mini Kit (Qiagen, Hilden, Germany). Superscript III Kit (Life Technologies) was applied for reverse transcription. cDNA was evaluated by quantitative PCR. Transcription was quantified and evaluated by RT‐PCR using the SYBR Green PCR Supermix kit (Bio‐Rad Laboratories, Hercules, CA, USA). Every procedure was carried out in triplicate. Real‐Time StatMiner (Integromics, Madrid, Spain) was used to assess gene expression.

### Transfections and RNA interference

Plasmids CDKL5‐pcDNA3.1 (CDKL5) and pcDNA3.1 (vector) were acquired from Shanghai GenePharma Co. Ltd. (Shanghai, China). U251 cells were seeded in six‐well plates 1 day before transfection. Transfection admixture was generated by adding 4 µg plasmid DNA and 3 µg TurboFect reagent (Fermentas, Glen Burnie, MD, USA) to DMEM/F12 without serum. The admixture was supplemented to the culture media, and the cells were further incubated for 6 h. In terms of siRNA transfection, U251 cells were transfected with 20 nmol control GL2 siRNA targeting the luciferase gene (shCDKL5#1: 5′‐CUA UGG AGU UGU ACU UAA AUU‐3′; shCDKL5#2: 5′‐GCA GAG UCG GCA CAG CUA UUU‐3′; siCtr 5′‐CGU ACG CGG AAU ACU UCG AUU‐3′) or siRNA oligonucleotides targeting CDKL5 using Lipofectamine RNAiMAX (Life Technologies).

### Cell survival

Cell survival was evaluated using the 3‐(4,5‐dimethylthiazol‐2‐yl)‐2,5‐diphenyl‐tetrazolium bromide (MTT) assay. Cells were seeded in 96‐well plates (5 × 10^4^ cells·mL^−1^). MTT assay was carried out 48 h after transfection. Cell survival was assessed by adding 10 μL MTT reagent to every well, and cells were further incubated for 4 h at 37 °C. The cells were examined using a microplate reader at 570 nm (Thermo Scientific, St. Louis, MO, USA). Every experiment was carried out three times independently.

### Cell migration

The Transwell assay was performed to evaluate cell migration. Cells were suspended in DMEM containing 1 mg·mL^−1^ mitomycin C. They were then seeded on the top chambers of 24‐well polycarbonate Transwell filters (Millipore, Bedford, MA, USA). Cells in DMEM containing 10% FBS were seeded to the bottom chambers. Cells at the top surface were scraped off after 48 h of incubation, whereas those at the bottom were fixed, stained and quantified.

The article "CDKL5 promotes proliferation, migration, and chemotherapeutic drug resistance of glioma cells via activation of the PI3K/AKT signaling pathway" was retracted in 2024. Reasons: plagiarized images; overlap with other authors' work; unreliable data; unreliable results or conclusions.

### Cell invasion

Transwell chambers that were covered with Matrigel were used to assess cell invasion. Transfected cells were seeded (1 × 10^5^ cells in each chamber) in the top chambers and incubated for 24 h. FBS (20%) served as a chemoattractant and was added to the chambers below. A cotton swab was used to eliminate noninvading cells on the top surface after incubation, whereas invading cells at the bottom were fixed with 100% methanol before staining with 1% crystal violet. Invading cells were quantified using a microscope, and six randomly selected visual fields were assessed for every assay.

### Cell cycle

Cells were starved for 12 h in preparation for synchronization before reactivation for 24 h with 10% FBS. Cells were fixed in 75% ethanol and treated with the Cell Cycle Detection Kit. A FACSCalibur flow cytometer (Beckman, San Francisco, CA, USA) was used to categorize the cells. flowjo software (Tree Star Inc., St. Louis, MO, USA) was used to assess the distribution of cell phase.

### Cell apoptosis

Apoptosis was assessed by flow cytometry (FC). The supernatant was eliminated after centrifugation for 5 min at 1000 ***g***. The sediment was resuspended with binding buffer. Propidium iodide and FITC/Annexin V were supplemented while the mixture was incubated for 10 min at 37 °C. A FACScan flow cytometer (Becton, Dickinson and Company, Franklin Lakes, NJ, USA) was used to evaluate fluorescence signals.

### *In vivo* malignant xenografts

Procedures related to animals were approved by the Ethical Committee of The First Affiliated Hospital of Dalian Medical University. The CDKL5 plasmid was constructed into the lentivirus vector LV‐3 (GenePharma). Stable cell lines with CDKL5 overexpression were selected with 4 μg·mL^−1^ puromycin incubation for 7 days. Nude male BALB/c mice aged 4 weeks were subcutaneously injected with approximately the stable clones of U251 cells (4–6 × 10^6^ cells), transfected with CDKL5, in their flanks regardless of the presence of infection. Mice were treated intraperitoneally with 5 mg·kg^−1^ cisplatin and 40 mg·kg^−1^ XL147 (Selleckchem, Houston, TX, USA) two times per week for 30 days . Every group consisted of five mice, which were executed after 30 days, and the malignancies were cut off and weighed.

### Western blotting

Lysis buffer (Beyotime, Wuhan, China) was applied to homogenize cell lysates and tissues, whereas protein quantification was carried out using the Bradford assay (Bio‐Rad). Protein evaluation was performed using SDS/PAGE. Tris/HCl polyacrylamide gels (8–15%; Bio‐Rad) were used to isolate proteins, which were moved to polyvinylidene fluoride membranes (Millipore). The blots were incubated overnight with primary antibodies [anti‐phosphoinositide 3‐kinase (PI3K), anti‐AKT, anti‐p‐PI3K (anti‐phosphorylated‐PI3K), anti‐p‐AKT, anti‐CDKL5, anti‐β‐actin; Cell Signaling Technology, Beverly, MA, USA] at 4 °C in TBS/Tween. Thereafter, the blots were incubated with secondary antibodies conjugated with horseradish peroxidase. Enhanced chemiluminescence plus detection reagent (Pierce, Rockford, IL, USA) was used to examine immunoreactive bands, which were assessed by the Omega 16ic Chemiluminescence Imaging System (Ultra‐Lum, Sacramento, CA, USA).

The article "CDKL5 promotes proliferation, migration, and chemotherapeutic drug resistance of glioma cells via activation of the PI3K/AKT signaling pathway" was retracted in 2024. Reasons: plagiarized images; overlap with other authors' work; unreliable data; unreliable results or conclusions.

### Statistical analysis

Results are displayed as mean ± SEM (standard error of the mean). Differences between groups were measured by two‐tailed, unequal‐variance Student’s *t*‐test and ANOVA before Tukey’s *post hoc* analysis. Statistical significance is indicated by *P* < 0.05.

## Results

### CDKL5 expression was promoted in glioma tissues

We examined CDKL5 in 27 normal cerebral specimens and gliomas to investigate the promising influence of CDKL5 on glioma generation and progression. CDKL5 transcription was noticeably upregulated in glioma tissues compared with that in normal tissues (Fig. 1A). Immunohistochemistry (IHC) and western blotting (WB) were performed to evaluate CDKL5. IHC revealed that CDKL5 translation was reinforced in glioma tissues in comparison with that in control tissues (Fig. 1B), which was confirmed by WB of fresh specimens (Fig. 1C,D). These findings suggested that CDKL5 expression was promoted in gliomas and that CDKL5 could be correlated to gliomas.

**Figure 1:** CDKL5 expression was enhanced in glioma specimens. (A) Quantitative RT‐PCR was used to examine CDKL5 transcription in glioma and normal cerebral specimens (*n* = 10). (B) Representative photomicrographs displaying CDKL5 expression in glioma and normal specimens (*n* = 8). Scale bar: 100 μm. (C, D) Representative immunoblots (C) and quantification of CDKL5 (D) in normal and glioma specimens (*n* = 9). Results are presented as means ± SEM. Student’s *t*‐test, **P < 0.01 versus normal group.

### CDKL5 enhanced migration invasion of glioma cells

We then examined the impact of CDKL5 on the migration and invasion of glioma cells. Noncoated Transwell chambers were used to evaluate the migration capability of U251 cells. It was shown that excessive CDKL5 expression remarkably promoted cell migration (Fig. 2A,B). The invasion capability of U251 cells was examined using polycarbonate Transwell filters coated with Matrigel. The number of U251 cells that invaded the Matrigel‐coated filters and arrived at the bottom surface of the membrane was elevated after transfection of CDKL5 in comparison with that of the blank control (Fig. 2C,D). In addition, CDKL5 overexpression significantly increased the expression of matrix metalloprotein 9 (MMP9) and matrix metalloprotein 2 (MMP2) in U251 cells (Fig. 2E). These findings suggested that CDKL5 enhanced the migration and invasion capability of U251 cells.

The article "CDKL5 promotes proliferation, migration, and chemotherapeutic drug resistance of glioma cells via activation of the PI3K/AKT signaling pathway" was retracted in 2024. Reasons: plagiarized images; overlap with other authors' work; unreliable data; unreliable results or conclusions.

**Figure 2:** CDKL5 enhanced migration and invasion of glioma cells. U251 cells transfected with empty vector or CDKL5 for 48 h. (A) Images displaying migration of U251 cells to the bottom surface. Scale bar: 100 μm. (B) Migrating U251 cells of various groups from five randomly selected visual fields visualized using a microscope. (C) Images displaying the invasion of U251 cells on the bottom surface. Scale bar: 100 μm. (D) Invading U251 cells of various groups from five randomly selected visual fields visualized using a microscope. (E) Representative immunoblots of MMP9 and MMP2 in U251 cells. Results are presented as means ± SEM. *n* = 3. Student’s *t*‐test, **P < 0.01 versus vector group.

### CDKL5 promoted proliferation and drug resistance of glioma cells *in vitro*

We explored the influence of CDKL5 on cell proliferation. The findings of the MTT assay proved that glioma cells with CDKL5 knockdown (KD) displayed remarkably reduced proliferation in comparison with that of the control group (Fig. 3A), whereas excessive CDKL5 expression promoted cell proliferation. The results of FC showed that the proportion of U251 cells in the S phase was noticeably elevated when CDKL5 was excessively expressed compared with control cells (Fig. 3B,C) and was obviously suppressed in CDKL5 KD cells.

**Figure 3:** CDKL5 reinforced drug resistance to β‐lap and glioma proliferation *in vitro*. U251 cells were transfected with CDKL5 plasmid (CDKL5) or CDKL5 siRNA (si‐CDKL5) for 48 h. (A) MTT assay was performed to examine cell survival. (B, C) Distribution of cell‐cycle phase was evaluated using FC. **P < 0.01 versus control group. (D–F) CDKL5 promoted drug resistance to β‐lap. U251 cells were transfected with CDKL5 plasmid (CDKL5) and supplemented with β‐lap. (D) MTT assay was performed to examine cell survival. (E, F) FC was performed to examine cell death. Results are presented as means ± SEM. *n* = 3. One‐way ANOVA, **P < 0.01 versus control group; ^#^ *P* < 0.05 versus β‐lap group.

We additionally explored whether CDKL5 regulated the malignancy counteraction activity of β‐lapachone (β‐lap), which served as an innovative malignancy‐counteracting agent that has been proved to stimulate various reactions of apoptosis in malignant cells. We evaluated cytotoxicity using the Cell Counting Kit‐8 and observed that cell survival was suppressed in the presence of β‐lap (Fig. 3D). Excessive CDKL5 expression clearly reduced the percentage of cell death. We also evaluated cell death using FC to better confirm the influence of CDKL5 on resistance to β‐lap. Supplementation with β‐lap evidently promoted cell death, and excessive CDKL5 expression prohibited this promotion (Fig. 3E,F). These findings indicated that CDKL5 participated in modulating the chemosensitivity to β‐lap in glioma cells.

The article "CDKL5 promotes proliferation, migration, and chemotherapeutic drug resistance of glioma cells via activation of the PI3K/AKT signaling pathway" was retracted in 2024. Reasons: plagiarized images; overlap with other authors' work; unreliable data; unreliable results or conclusions.

### CDKL5 promoted stimulation of the PI3K/AKT axis in glioma cells

The PI3K/AKT axis participates in the modulation of cell proliferation and invasion 21. We subsequently explored the impact of CDKL5 on the phosphorylation of the PI3K/AKT axis using WB. As shown in Fig. 4, CDKL5 overexpression obviously increased the phosphorylation level of PI3K, AKT and GSK3, whereas CDKL5 KD significantly inhibited the phosphorylation level of PI3K, AKT and GSK3. These findings proved that CDKL5 reinforced the stimulation of the PI3K/AKT axis in glioma cells.

**Figure 4:** CDKL5 reinforced stimulation of the PI3K/AKT axis in glioma cells. (A–D) Representative immunoblots (A) and quantification of phosphorylation of PI3K (B), AKT (C) and GSK3β (D) in U251 cells after transient transfection with CDKL5 plasmid (CDKL5) or empty vector (Vector) for 48 h. Results are presented as means ± SEM. *n* = 3. **P < 0.01 versus vector group. (E–H) Representative immunoblots (E) and quantification of phosphorylation of PI3K (F), AKT (G) and GSK3β (H) in U251 cells after transient transfection with CDKL5 siRNA (si‐CDKL5) or negative control (NC) for 48 h. Results are presented as means ± SEM.* n* = 3. Student’s *t*‐test, **P < 0.01 versus NC group.

### CDKL5 quickened glioma generation through PI3K/AKT axis *in vivo*

Nude male BALB/c mice were injected with U251 cells with CDKL5 plasmid in the flanks, and malignancies were weighed 30 days later to explore whether CDKL5 reinforced glioma proliferation *in vivo*. PI3K inhibitor XL147 significantly reduced the CDKL5‐induced phosphorylation level of AKT *in vivo* (Fig. 5A). Mice that were injected with U251 cells with CDKL5 plasmid exhibited noticeably larger malignancies in comparison with those in the vector, which were attenuated via prohibition of the PI3K/AKT axis (Fig. 5B–D). Moreover, IHC evaluation of Ki67, a biomarker of growth, was carried out in malignant xenograft tissues. Excessive expression of CDKL5 remarkably elevated Ki67 concentration, which was counteracted via prohibition of the PI3K/AKT axis (Fig. 5E). These results indicated that CDKL5 promoted glioma carcinogenesis via stimulation of the PI3K/AKT axis.

The article "CDKL5 promotes proliferation, migration, and chemotherapeutic drug resistance of glioma cells via activation of the PI3K/AKT signaling pathway" was retracted in 2024. Reasons: plagiarized images; overlap with other authors' work; unreliable data; unreliable results or conclusions.

**Figure 5:** CDKL5 quickened glioma generation through the PI3K/AKT axis *in vivo*. Mice were subcutaneously injected with stable U251 cells with CDKL5 plasmid (CDKL5) and administered with cisplatin and PI3K/AKT suppressor XL147 (CDKL5 + CP + XL147). (A) Representative immunoblots of p‐AKT in tumor tissues. (B, C) Representative images of malignancies (B) and quantification of malignancy volume (C) and weight (D) 4 weeks after subcutaneous xenografting. (E) Representative IHC images of Ki67 in slices. Scale bar: 40 μm. Results are presented as means ± SEM. *n* = 5. One‐way ANOVA, *P < 0.05 versus vector group; ^#^ *P* < 0.05 versus CDKL5 group.

## Discussion

Our research showed that CDKL5 expression was promoted in glioma specimens in comparison with that in normal specimens. The activity of CDKL5 in glioma cells was studied by excessive expression and KD assays. We discovered that excessive CDKL5 expression reinforced drug resistance, migration, proliferation and invasion in glioma cells, whereas CDKL5 KD resulted in the opposite effects. CDKL5 enhanced the stimulation of the PI3K/AKT axis, which subsequently participated in glioma generation. Collectively, our findings reveal that CDKL5 can modulate glioma proliferation, and that the PI3K/AKT axis participates in this reaction. The results of this research throw light upon both the influence of CDKL5 on gliomas and strategies of glioma therapy.

Gliomas are one of the most fatal malignancies in the central nervous system, with glioblastoma being the most common form, which features poor median survival of 15 months and extreme aggressiveness 22, 23. Despite rapid progress in glioma diagnosis and therapy, the 5‐year survival has not improved significantly, emphasizing the need to recognize and investigate the molecular etiology of glioma generation 24, 25, 26. In the past 10 years, genetic damage has been discovered in patients suffering from neurological diseases, which appear as an early attack of usually refractory epilepsy, mental retardation and suppressed motor regulation 27, 28. Because mutations in CDKL5 have a noticeable influence on cerebral activities, most studies aim to study the influence of this kinase on neurons, but little has been revealed in terms of its effect on growing cells 29, 30. Almost no information has indicated that CDKL5 participates in cell growth 31. Excessive expression of CDKL5 triggers cell cycle arrest of neuroblastoma cells, whereas CDKL5 suppression via RNA interference or aimed gene disturbance was shown to promote the incorporation of bromodeoxyuridine 32, 33. Nevertheless, understanding of the effect of CDKL5 on gliomas is insufficient. Our research has revealed some novel aspects. We proved that CDKL5 expression was reinforced in glioma tissue samples and that CDKL5 enhanced glioma migration and invasion. Next, elevation in CDKL5 expression was shown to stimulate drug resistance and cell growth not only *in vivo* but also *in vitro*. Furthermore, CDKL5 KD stimulated counteracting effects on malignancy growth. These findings can assist us in understanding the etiology of the oncogenic effect of CDKL5 and alter our perspective of its impact as a candidate treatment agent. *In vivo* findings indicated that CDKL5 enhanced glioma generation by stimulating the PI3K/AKT axis.

The article "CDKL5 promotes proliferation, migration, and chemotherapeutic drug resistance of glioma cells via activation of the PI3K/AKT signaling pathway" was retracted in 2024. Reasons: plagiarized images; overlap with other authors' work; unreliable data; unreliable results or conclusions.

The PI3K/AKT axis is related to metastasis and glioma development 34, 35, 36, 37, 38. Previous research has shown that SRPK1 enhanced metastasis and vessel generation in gliomas via the PI3K/AKT axis 39. As a conventional Chinese herbal medicine, shikonin was demonstrated to suppress invasion and migration of glioblastoma cells by targeting the PI3K/AKT axis 40, 41. We discovered that excessive CDKL5 expression promoted the phosphorylation of PI3K and AKT, which was prohibited by CDKL5 KD, indicating that CDKL5 stimulated the PI3K/AKT axis. As a serine/threonine kinase, CDKL5 may activate PI3K via interacting with PI3K. Moreover, we found that prohibition of this axis attenuated the effect of excessive CDKL5 expression on glioma generation *in vivo*. The results of our research suggested that CDKL5 reinforces the generation of gliomas through the PI3K/AKT axis.

## Conclusions

In summary, our research demonstrated that CDKL5 expression is reinforced in gliomas, and that it affects the proliferation, migration, drug resistance and invasion of glioma cells. Furthermore, CDKL5 enhances the generation of gliomas *in vivo* by stimulating the PI3K/AKT axis. This research emphasizes the promising effect of CDKL5 on the assessment of clinical outcome and treatment application of gliomas.

## Conflict of interest

The authors declare no conflict of interest.

## Author contributions

ZJ and HW conceived the study and designed the experiments. ZJ, TG and HW contributed to the data collection, performed the data analysis and interpreted the results. ZJ wrote the manuscript. ZJ and HW contributed to the critical revision of the article. All authors read and approved the final manuscript.
